The article "Motion Accuracy of Pneumatic Stepper Motor-Driven Robotic System Developed for MRI-Guided High-Intensity Focused Ultrasound Treatment of Prostate Disease" was published in 2024. Journal: Appl Bionics Biomech.

# Motion Accuracy of Pneumatic Stepper Motor-Driven Robotic System Developed for MRI-Guided High-Intensity Focused Ultrasound Treatment of Prostate Disease

**DOI:** 10.1155/2024/5556537

**Published:** 2024-05-10

**Authors:** Hyunkwan Seo, Sung Kwan Hwang, Hee-Won Kim, Kyu Chan Lee

**Affiliations:** ^1^Gachon Biomedical Convergence Institute, Gachon University Gil Medical Center, Incheon, Republic of Korea; ^2^Medrobotics, Seongnam-si, Gyeonggi-do, Republic of Korea; ^3^Coretech Co., Ltd., Seongnam-si, Gyeonggi-do, Republic of Korea; ^4^Department of Radiation Oncology, Gil Medical Center, Gachon University College of Medicine, Incheon, Republic of Korea

## Abstract

The latest advancement in high-intensity focused ultrasound (HIFU) treatment technology integrates magnetic resonance imaging (MRI) guidance for precise treatment of prostate disease. As conventional electromagnetic motors are not applicable for utilization within MRI scanners, we have developed a prototype robotic system driven by pneumatic stepper motors to control the movement of the HIFU transducer within an intrarectal probe during MRI-guided HIFU treatment procedures. These pneumatic stepper motors were constructed entirely from MRI-compatible plastic materials. Assessment of the robotic system's MRI compatibility was conducted utilizing a 3.0T MRI scanner, revealing no discernible MRI image distortion with a minor decrease in the signal-to-noise ratio (2.8%) during the motor operation. The robotic system enabled the transducer to move inside the probe with two degrees of freedom, allowing both linear and rotational motion. The positional accuracy of the transducer movement was assessed, yielding ±0.20 and ±0.22 mm accuracies in the forward and backward linear movements, respectively, and ±0.79° and ±0.74° accuracies in the clockwise and counterclockwise rotational motions, respectively. Emulation of authentic HIFU procedures involved creating a two-dimensional array of thermal lesions in a tissue-mimicking phantom, achieving positional accuracy within ±1 mm for the generated HIFU focal spots. The prototype robotic system incorporating pneumatic stepper motors fabricated entirely from MRI-compatible plastic materials has demonstrated the requisite positional accuracy necessary for effective HIFU treatment of prostate disease, indicating substantial promise for future clinical application.

## 1. Introduction

High-intensity focused ultrasound (HIFU) systems conically focus on ultrasound beams with frequencies ranging from hundreds of kilohertz to megahertz to generate high-intensity focal points in tissues and induce heat. This, in turn, results in coagulative necrosis in the tissue, which is the main concept utilized in treatments for various benign or malignant tumors [1–5]. HIFU treatment is a noninvasive procedure with no harmful radiation effects [6]. If a lesion is accurately targeted, the surrounding healthy tissues remain unharmed, leading to fewer side effects [7]. Moreover, HIFU treatment is an outpatient procedure with a short recovery time and is a patient-friendly treatment that facilitates a better quality of life [8]. The ultrasound-guided transrectal HIFU technique has been utilized in prostate cancer treatment for over 20 years [9]. However, the ultrasound-guided method cannot accurately monitor the spatial distribution of the lesion and the intensity of the HIFU at the acting point. It also has an interference problem between the HIFU and monitoring signals. In the case of prostate treatment, there is a risk of incomplete treatment or harm to normal tissues due to side effects, such as edematous deformation, during or immediately after the procedure [10]. Recently, a magnetic resonance imaging (MRI)-guided HIFU system has been introduced to reduce complications that may occur during prostate treatment utilizing ultrasound-guided HIFU [11]. With excellent soft tissue contrast, an MRI-guided HIFU system can precisely locate tumors and monitor the formation of the HIFU focal spot, an area of denaturation in tissue, and treated volume in real time. In addition, tissue temperature can be measured during the procedure by utilizing the temperature-imaging capability of MRI [12, 13].

The article "Motion Accuracy of Pneumatic Stepper Motor-Driven Robotic System Developed for MRI-Guided High-Intensity Focused Ultrasound Treatment of Prostate Disease" was published in 2024. Journal: Appl Bionics Biomech.

In MRI-guided HIFU therapy, it is an absolute prerequisite that all components and parts of the entire HIFU system do not interfere with the magnetic field and operate independently of it. Because electromagnetic motors are neither magnetic resonance (MR)-compatible nor MR-safe, other types of motors, such as hydraulic, piezoelectric, and pneumatic motors, should be considered. Among these options, pneumatic motors offer excellent MR compatibility, with a negligible change of a signal-to-noise ratio (SNR) of MRI images [14]. Though pneumatic motors may have a poor ability for exact positioning control owing to the elastic or resilient compressibility of air, several studies have reported achieving precise motion control utilizing the step motor principle in pneumatic motors in the medical field [15–18]. Stoianovici et al. [15] developed the first pneumatic stepper motor and applied it to an MR-compatible robot performing transperineal percutaneous needle access to the prostate for prostate brachytherapy. After Stoianovici's first development of the pneumatic stepper motor applied to the MR system, smaller, simpler, and easier-to-use prototypes of pneumatic stepper motors have been studied. Sajima et al. [16] developed a compact, easy-to-manufacture pneumatic stepping actuator comprising three linear gears and a rotary gear. Chen et al. [17] developed the motor using a LEGO® cylinder, and the gearbox allows flexible gear ratio adjustment. Groenhuis and Stramigioli [18] developed five pneumatically driven linear and rotary stepper motors utilizing rapid prototyping techniques such as 3D printing and laser cutting.

The article "Motion Accuracy of Pneumatic Stepper Motor-Driven Robotic System Developed for MRI-Guided High-Intensity Focused Ultrasound Treatment of Prostate Disease" was published in 2024. Journal: Appl Bionics Biomech.

Convinced by the reports on developing precise and compact pneumatic stepper motors, we designed and developed a metal-free MR-compatible pneumatic stepper motor for the robotic device in our transrectal HIFU system to treat prostate disease. We introduced a potentiometer to achieve secure position control, creating a closed-loop feedback system. Our pneumatic stepper motors were manufactured with a 3D printer and polylactic acid (PLA), a plastic material commonly employed in 3D printing, which offers several advantages, including fast prototype production, low cost, lightweight properties, and ease of replication. We then applied these pneumatic motors to the MRI-guided transrectal HIFU system that we are developing, evaluating the positional accuracy of the transducer and the stepwise scanning ability of the transrectal HIFU robot system with the same setup as the actual HIFU procedure. The goal of the geometrical positioning accuracy of the HIFU focal spot for our system was to be within ±1 mm in accordance with the guidelines of the Ministry of Food and Drug Safety (MFDS) in South Korea.

## 2. Materials and Methods

### 2.1. Transrectal HIFU System

#### 2.1.1. HIFU Transducer

Developed for prostate treatment, the HIFU transducer assembly (KEMSTI Co., Ltd., South Korea) has a diameter of 2.5 cm, making it suitable in size for a transrectal HIFU system, and contains two MR-compatible rounded concave transducers with different focal lengths, facing back to each other, enabling selective utilization depending on the depth of the tumor. Considering the distance between the transducer and the tumor when inserted into the rectum, one side was operated at a frequency of 4.79 MHz with a focal length of 30 mm, and the other was operated at a frequency of 3.36 MHz with a focal length of 45 mm.

#### 2.1.2. Probe Design

The transducer assembly was mounted inside the probe designed to be inserted into the rectum to irradiate the human prostate with HIFU. The shape of the probe housing the transducer is depicted in Figure 1. The probe head, the distal end of the probe, was designed to have an outer diameter of 35 mm to be inserted into the human rectum. Considering the prostate length along the patient's rectal axis (the *Z*-axis), the probe head was designed to be 105 mm long and had an open window through which the transducer could irradiate HIFU toward the target. The transducer could be moved within the open window of the probe head with two degrees of freedom (DOF): one rotational motion with an ablation angle of 90° and one linear motion with an ablation length of 60 mm. This enables comprehensive scanning of the entire prostate. The probe head was connected to a 70-mm-long neck, tapered from the head, and positioned at the sphincter of the human rectum such that the head could reach the prostate. A spur gear and a rack gear were integrated into the cylindrical body of the probe, allowing it to be connected to an external actuator that generated both the rotational and linear motions of the transducer. The probe's body was made of polyoxymethylene, and the gears were made of monomer-cast nylon. Both the materials and some aluminum and rubber parts were MR-compatible. All the parts were held together with reinforced nylon screws.

The article "Motion Accuracy of Pneumatic Stepper Motor-Driven Robotic System Developed for MRI-Guided High-Intensity Focused Ultrasound Treatment of Prostate Disease" was published in 2024. Journal: Appl Bionics Biomech.

#### 2.1.3. Degassed Water and Cooling System

The probe head was covered with an ultrasound probe cover (PC-SIL-02; Innolatex, Sdn. Bhd., Malaysia), a sterilized disposable product made of natural rubber latex. The cover was filled with water as an ultrasound transmission medium between the transducer and the target tissue. The water medium must be degassed with a dissolved oxygen concentration ≤5 ppm to prevent bubble formation in the HIFU beam path, which reduces the cauterization effect. Degassed water was cooled with an external heat exchanger and circulated to cool the rectal wall.

### 2.2. Pneumatic Stepper Motor-Driven Robotic Device

#### 2.2.1. Design Consideration of Robotic Device

The robotic device is designed to accommodate the patient's dorsal recumbent position on the MRI couch. In this posture, where the patient's legs are folded onto the treatment couch, the distance from the couch to the anus (referred to as “height” hereinafter) measures ∼6 cm for an adult patient. The robotic device should position the probe at this height, ensuring precise alignment with the patient's anatomy to enable smooth and controlled insertion into the rectum. Furthermore, the device's dimensions should be much smaller than those of the couch to facilitate easy and secure mounting of the robotic unit onto the couch.

#### 2.2.2. Motor Design and Working Principle

To ensure compatibility with the strong magnetic field of MRI, all parts of the pneumatic motor were made of polylactic acid (PLA), a plastic made with a 3D printer. The developed pneumatic motor was a rotational stepper motor with dimensions of 61 × 61 × 34 mm. The motor features a radially placed four-cylinder configuration that is actuated by sequential pneumatic pulses (Figure 2 for the SolidWorks design and Figure 3(a) for the physical version). Inspired by the design principle of the Groenhuis R-80 motor [18], this configuration effectively converts axial piston motion into rotational motion.

The article "Motion Accuracy of Pneumatic Stepper Motor-Driven Robotic System Developed for MRI-Guided High-Intensity Focused Ultrasound Treatment of Prostate Disease" was published in 2024. Journal: Appl Bionics Biomech.

The pneumatic stepper motor comprises four cylinders, two pistons, and a geared axle. Compressed air is sequentially supplied to the four cylinders via respective individual pneumatic tubes. As air pressure is sequentially transmitted to each cylinder, it imparts force onto the pistons within the motor, inducing linear oscillations and generating a series of discrete rotational steps on the geared axle (Figure 4). The internal gear of the motor had nine teeth, advancing by one tooth after every four pneumatic pulse outputs. To enhance the output torque, the motor was coupled to a planetary gearbox with dimensions of 61 × 61 × 32 mm (Figure 3(b)), enabling it to operate at a gear ratio of 64 : 1. Consequently, 64 × 9 × 4 input pulses are required for one full rotation of its axis.

#### 2.2.3. Design of Robotic Device

An MRI-compatible robotic system was constructed by integrating a HIFU probe with three pneumatic stepper motors (Figure 5). The proximal end of the probe, located outside of the patient's body, was securely fastened to the robot's probe holder designed to fit into a groove (Figure 1(b)) on the probe's surface. Motors 1 and 2 control the *Z*-axis and *Φ*-axis movements of the transducer within the probe head, respectively. Meanwhile, Motor 3 oversees the *Z*-axis movement of the entire assembly, which includes the probe, probe holder, Motor 1, and Motor 2. Because the developed pneumatic motors are rotational stepper motors, we achieved linear motion along the *Z*-axis for both the transducer and the entire assembly by utilizing a rack and pinion mechanism. In this configuration, a rack attached to the probe body engages with a pinion gear, which is driven by Motor 1 to control the *Z*-axis movement of the transducer. Similarly, Motor 3 is also connected to an additional rack, enabling it to control the *Z*-axis motion of the entire assembly. For the transducer's rotational motion, one rotation of the motor axis rotates the transducer by approximately one revolution. By contrast, for the linear motion, one rotation of the motor axis moves the transducer by 25 × 3.14 mm.

The horizontal placement height of the probe on the treatment couch is typically positioned at ∼6 cm, corresponding to the average height of the anus and rectum when a male adult patient is in a treatment position on the couch. Moreover, this height can be manually adjusted along the *Y*-axis using height adjustment knob, as depicted in Figure 5(b), to accommodate variations in individual patients' anal and rectal heights. In addition, the probe holder was designed to rotate freely around an axis parallel to the *X*-axis and passing through the center of the height adjustment knob (Figure 5(b)). This structural design facilitates accommodation for abrupt changes in the insertion angle, represented as *Θ* in Figure 5(b), during the insertion process of the probe into the rectum via the anus, in response to individual variations in the anorectal angle. Anatomically, although individual variations may exist, the rectum and anus typically form an angle of ∼90°, known as anorectal angle, when observed in the sagittal plane through lateral projection. Therefore, the probe is inserted into the anus, advanced a few centimeters, and then angled appropriately to align with the direction of the rectum as it passes through the anal sphincter, facilitating further insertion into the rectum. Guided by the MRI image, the probe is manually positioned just above the prostate according to each patient's anatomy. Subsequently, it is secured in place utilizing the height adjustment knob. Once inserted, the natural contraction and tightening of the sphincter muscle around the probe neck help prevent movement of the probe throughout the procedure, providing additional stability.

The article "Motion Accuracy of Pneumatic Stepper Motor-Driven Robotic System Developed for MRI-Guided High-Intensity Focused Ultrasound Treatment of Prostate Disease" was published in 2024. Journal: Appl Bionics Biomech.

During the HIFU procedure for the treatment of prostate disease, the probe remains fixed in the rectum, while only the transducer is moved along the *Z*- and *Φ*-axes within the probe, utilizing Motors 1 and 2. Motor 3 may be utilized, if required, to initially adjust the probe's position along the *Z*-axis relative to the robotic device's baseplate, based on the patient's posture. Nevertheless, it does not participate in positioning the transducer during the procedure. The baseplate of the robotic device, with dimensions of 20 cm in width and 39 cm in length, was much smaller than the MRI couch. This compact size ensures convenient and secure device mounting onto the couch. All components employed to integrate the pneumatic stepper motors to the HIFU probe, like the pneumatic motors, were made of PLA, a 3D-printed plastic material compatible with MRI.

A closed-loop system with position feedback was implemented with three rotary potentiometers (6639S; Bourns Inc., USA) to monitor and control the three movements actuated by the motors. Because of the utilization of potentiometers, our robotic system was classified as MRI-conditional according to the American Society for Testing and Materials (ASTM) classification (F2503) for MRI.

The article "Motion Accuracy of Pneumatic Stepper Motor-Driven Robotic System Developed for MRI-Guided High-Intensity Focused Ultrasound Treatment of Prostate Disease" was published in 2024. Journal: Appl Bionics Biomech.

#### 2.2.4. External HIFU Robotic System Controller

While the robotic device is positioned inside the MRI scanner, certain equipment, such as an air compressor and electromagnetic valves incompatible with MRI, must be located outside the MRI bore. Consequently, the pneumatic stepper motors that rely on air pressure control must be controlled externally.

To produce compressed air for the pneumatic stepper motor, a commercial air compressor (DC886; KOLAVO, South Korea) with a 4-horsepower motor, a 17-L aluminum tank, a pressure of 0.3–12 MPa, and a flow rate of 250 L/min was utilized. The air compressor, which utilizes a brushless motor with a permanent magnet and steel parts made of ferromagnetic materials, was placed outside the MRI room. The air compressor was initially set to 1.00 MPa. Subsequently, the pressure was further adjusted to 0.55 MPa utilizing a pressure regulator before reaching the solenoid valves. The sequential delivery of pressurized air to the four cylinders of each motor was controlled by solenoid valves, which cannot be utilized inside the MRI bore. The solenoid valves were therefore placed in an external robotic system controller (Figure 6) 5 m away from the MRI bore, and the three pneumatic stepper motors of the robotic system were connected to the valves utilizing twelve 5-m-long plastic pneumatic tubes (four cylinders × three motors).

The Arduino Uno board in the external robotic system controller operates the electromagnetic solenoid valves. The analog output signals of the potentiometers were also connected to an analog-to-digital converter (ADC) of the Arduino Uno board as an input to provide the positional information of the transducer. Arduino Uno sends a signal to the signal generator (Jeisys Medical Inc., South Korea), which applies a radio frequency signal to the transducer to generate the ultrasound. The controller communicates with the personal computer (PC) via the recommended standard 232 protocol. Scanning pathways of the transducer and firing sequence of the HIFU application were programed and executed utilizing computer software (Arduino 1.8.13). Sonication parameters, such as frequency, acoustic power, pulse duration, duty cycle, and sonication time, were also controlled with the Arduino 1.8.13 software.

### 2.3. MRI Compatibility

The MRI compatibility assessment of the robotic device was conducted utilizing a 3.0T MRI scanner (MAGNETOM Vida, Siemens Healthcare, Erlangen, Germany). MRI images were acquired employing a 64-Channel Head/Neck coil with a cylindrical phantom (Siemens Healthcare GmbH, Germany) filled with distilled water doped with 3.75 g NiSO_4_ × 6H_2_O, 5 g NaCl per 1,000 g H_2_O. The robotic device was positioned within the MRI bore (Figure 7), while the external controller, mounted in a rack, was placed 5 m away inside the MRI room, and the air compressor was situated outside the room. The evaluation utilized images obtained from a T1-weighted gradient echo (T1 GRE) sequence under three distinct conditions: (1) the MR phantom only in the MRI bore served as a baseline control image; (2) the presence of the robot device connected to an external controller in the MRI bore; and (3) the operation of the robotic device, involving the activation of Motors 1 and 2 along with their corresponding potentiometers. For each condition, a qualitative visual evaluation was conducted by subtracting the test MRI images (condition 2 or 3) from the baseline control image (condition 1) to identify and analyze any discrepancies or variations. MRI compatibility was quantitatively evaluated by measuring the SNR. SNR was defined as the ratio of the mean intensity and standard deviation (SD) within a 20 × 20 pixel region located at the center of the phantom image. Each pixel had a scale of 0.9375 mm.

The article "Motion Accuracy of Pneumatic Stepper Motor-Driven Robotic System Developed for MRI-Guided High-Intensity Focused Ultrasound Treatment of Prostate Disease" was published in 2024. Journal: Appl Bionics Biomech.

### 2.4. Evaluation of Motion Accuracy

To replicate the actual HIFU procedure in our motion accuracy experiments, we connected the pneumatic stepper motors and the solenoid valves within the external controller via 5-m-long pneumatic tubes, attached the HIFU probe to the robotic device, and externally controlled the transducer's motion within the probe utilizing a PC. For prostate treatment, we defined a stepwise scanning interval of 3 mm along the *Z*-axis and 8.6° in the *Φ*-axis direction, particularly when utilizing a transducer with a 30-mm focal length. We chose an 8.6° rotation angle because it corresponds to a 3-mm displacement of the lesion on a plane perpendicular to the HIFU beam, positioned 20 mm away from the center of the transducer surface. These adjustments were made to account for the fact that, during HIFU procedures, lesions tend to form at distances closer than the geometric focal length because of various factors, such as changes in the energy absorption characteristics of tissues during the HIFU scan [19].

Subsequently, we evaluated the transducer's motion accuracy by causing it to move with these defined spatial intervals and subsequently assessing its actual motions. The potentiometer ADC value change corresponding to a unit displacement in both the *Z*- and *Φ*-axis directions had been predetermined through calibration. For evaluating the linear motion accuracy along the *Z*-axis, Motor 1 was pulsed until an ADC value change corresponding to a 3-mm transducer movement was achieved, followed by the measurement of the actual transducer displacement. The displacement error was defined as the difference between the actual transducer displacement and the intended 3 mm. Similarly, to assess the rotational angular motion accuracy along the *Φ*-axis, Motor 2 was pulsed, inducing an ADC value change equivalent to an 8.6° rotation of the transducer, and the actual angular displacement of the transducer was measured. The angular displacement error was defined as the difference between the actual angular displacement of the transducer and the intended 8.6°.

The article "Motion Accuracy of Pneumatic Stepper Motor-Driven Robotic System Developed for MRI-Guided High-Intensity Focused Ultrasound Treatment of Prostate Disease" was published in 2024. Journal: Appl Bionics Biomech.

### 2.5. Evaluation of Lesion Formation in Human Tissue-Mimicking Phantom

In the human body, the prostate tumors typically manifest with a size of one cubic centimeter or larger. Considering that each HIFU focal spot induces a coagulative necrosis lesion in live human tissue with a volume of several cubic millimeters, it is essential to fire HIFU focal spots at millimeter intervals to ensure effective cauterization of the target tumor. As the size of the tumor to be treated varies, we evaluated the capability of the robotic system to generate lesions in an array pattern of various sizes in a tissue-mimicking phantom. Bovine serum albumin (BSA) phantom was fabricated in the laboratory to mimic the HIFU energy absorption in human tissue with the recipe proposed by Lafon et al. [20]; the weight/volume concentration of the BSA was 5%. Our research collaborators, Song et al. [21], also employed the BSA phantom made with the same recipe in their HIFU study published in 2013. Lafon et al. [20] reported that the BSA gel phantom exhibited a sound speed of 1,544 m/s and a density of 1,044 kg/m^3^, both comparable to those of soft tissues, while its attenuation coefficient measured 0.013 Np/cm/MHz for 5% BSA, which was significantly lower than that observed in soft tissues. Nonetheless, the disparity in the attenuation coefficient does not impact the evaluation of the mechanical motion in our robotic system. In addition, Lafon et al. [20] reported that the BSA phantom's thermal properties are expected to be similar to those of egg-white polyacrylamide gel phantom, which has been previously characterized with a specific heat of 4,270 J/kg/°C and a thermal conductivity of 0.59 W/m/°C [22], values comparable to those of water. The BSA phantom is a transparent gel that forms a visible whitish opaque lesion when exposed to temperatures above 58°C due to BSA protein denaturation [20]. When sufficient HIFU energy is applied with appropriate focusing, an area of high temperature above 60°C is generated, called the HIFU focal spot. This focal spot can be easily recognized by the naked eye in the BSA phantom and can be visualized in some imaging modalities such as ultrasound or MRI.

The article "Motion Accuracy of Pneumatic Stepper Motor-Driven Robotic System Developed for MRI-Guided High-Intensity Focused Ultrasound Treatment of Prostate Disease" was published in 2024. Journal: Appl Bionics Biomech.

The experimental setup adopted to irradiate HIFU in the BSA phantom is depicted in Figure 8. The probe head was covered with a silicone probe cover filled with degassed water, and the probe and the probe cover were placed near the phantom. The degassed water was circulated through two-way hoses between the probe and the water circulator with a heat exchanger and a degassing device.

The generation of a two-dimensional (2D) array of HIFU focal spots on the BSA phantom was accomplished by incrementally moving the transducer within the probe head along two DOF: the *Z*- and *Φ*-axes, while maintaining the probe stationary. The movement of the transducer followed a zigzag raster scanning pathway, as illustrated in Figure 9, which represents a 3 × 3 array configuration. Motor 2 induced rotational motion of the transducer along the *Φ*-axis, resulting in lesion arrays in the *X*-axis direction within the *X*–*Z* plane, while Motor 1 controlled the transducer's movement along the *Z*-direction. At each point along the scanning path, HIFU energy was emitted from the transducer with a focal length of 30 mm, with HIFU pulse cycles of 250 ms “on time” and 50 ms “off time” for 6 s at an acoustic power of 35 W.

## 3. Results

### 3.1. MRI Compatibility

Visual inspection of the test MRI images acquired under the “robot connected” (Figure 10(b)) and “robot in operation” (Figure 10(c)) conditions revealed no discernible noise or image distortion compared to the control image (Figure 10(a)). The subtraction images (Figures 10(d) and 10(e)), derived by subtracting each test image from the control image, exhibited no significant distinctions.

The SNR value was calculated based on the mean intensity and SD of the MRI images acquired under the three distinct conditions (Table 1). In comparison to the “phantom only” image, the “robot connected” condition exhibited a 2.5% decrease in SNR, while the “robot in operation” condition showed a decrease of 2.8%.

### 3.2. Positional Accuracy

The linear displacement error as the transducer moves along the *Z*-axis, driven by Motor 1, with 3-mm step increments is depicted in Figure 11(a). The transducer executed ten forward linear steps, followed by an equal number of backward steps.  Figure 11(b) illustrates the angular displacement error during the transducer's rotation along the *Φ*-axis. This rotation was driven by Motor 2 with 8.6° step increments, involving ten clockwise (CW) rotational steps, followed by a reversal in direction with counterclockwise (CCW) rotational steps. In both linear and rotational motions, significant larger errors of −1.8−2.2 mm for linear motion and −4.4°−4.7° for rotational motion were observed during the 1st and 11th steps, compared to the errors during the other steps. These particular steps corresponded to instances where the direction of the transducer's movement changed. The backlash created between the mated gears is the main cause of the larger error when changing the direction in both linear and rotational motions. A software compensation method was applied to compensate for the backlash offset when the motor changed direction by adding one more step in the changed direction and taking it back in one step. The backlash compensation was effective, resulting in displacement errors during those particular steps becoming indistinguishable from errors during the other steps for both linear and rotational motions (Figures 11(c) and 11(d)).

The article "Motion Accuracy of Pneumatic Stepper Motor-Driven Robotic System Developed for MRI-Guided High-Intensity Focused Ultrasound Treatment of Prostate Disease" was published in 2024. Journal: Appl Bionics Biomech.

To quantitatively measure the positional accuracy of transducer movement, we plotted error distributions for four different movements, each obtained by sampling 40 times (Figure 12). These four distinct motions correspond to those presented in Figure 11: forward and backward linear movements along the *Z*-axis with 3-mm step increments, as well as CW and CCW rotational movements along the *Φ*-axis with 8.6° step increments. Each of the four distributions was fitted utilizing a Gaussian function to determine the mean, standard error of mean (SEM), and standard deviation (SD), summarized in Tables 2 and 3 for the linear and rotational motions, respectively. The deviation of the mean of the distribution from the zero error reflects the calibration error, while the SD indicates the positional accuracy of each motion.

The mean of the error distribution for forward linear motion along the *Z*-axis is consistent with the zero error within the SEM. Furthermore, the mean of the error distribution for backward linear motion along the *Z*-axis is 0.13 mm smaller than the zero error. The change in the ADC value of the potentiometer output, corresponding to a unit displacement of the transducer, must be periodically calibrated due to the shift in the mean of the error distribution over time, attributed to the aging of the robotic device. Similarly, the mean of the angular error distribution in the CW direction along the *Φ*-axis was 0.18° greater than the zero error, and the mean of the angular error distribution in the CCW direction along the *Φ*-axis was 0.13° greater than the zero error. As with linear motion, rotational motion should be periodically calibrated based on the shift in the mean of the angular distribution from the zero error.

The measured positional accuracies of the linear motions meet the focal positional accuracy goal of our HIFU system, which is set within 1 mm (Table 2). As for rotational motions, the angular positional accuracies were less than 0.80° (Table 3). A 0.80° rotation error of the transducer results in a position error of 0.42 mm at a focal length of 30 mm and 0.63 mm at a focal length of 45 mm, as determined by the relation Δ*l*=*r* · tan(Δ*θ*), where Δ*l* is the position error in the plane perpendicular to the HIFU beam at the focal length, *r* is the focal length, and Δ*θ* is the rotation error. Consequently, the measured positional accuracy of the robotic system meets the focal position accuracy goal of our HIFU system for treating prostate disease, both in the linear and rotational motions.

The article "Motion Accuracy of Pneumatic Stepper Motor-Driven Robotic System Developed for MRI-Guided High-Intensity Focused Ultrasound Treatment of Prostate Disease" was published in 2024. Journal: Appl Bionics Biomech.

### 3.3. Verification through Creation of Lesions in Human Tissue-Mimicking Phantom

With the robotic system, we successfully generated five different array patterns of HIFU thermal lesions, with the HIFU focal spots clearly visible as opaque whitish color to the naked eye in the BSA phantom (Figure 13), demonstrating the capability of the robotic system to target tumors of various sizes. In the array patterns presented in Figure 13, the left–right direction corresponds to the transducer's rotational motion along the *Φ*-axis, while the up–down direction corresponds to the linear motion along the *Z*-axis. We utilized a transducer with a focal length of 30 mm, and the rotation angle interval was set to maintain the same lesion spacing as in the linear motion. The five array patterns are as follows: (a) a 3 × 3 array with 2-mm spacing for linear movement and 5.7° spacing for rotational movement, (b) a 3 × 3 array with 3-mm spacing for linear movement and 8.6° spacing for rotational movement, (c) a 3 × 3 array with 1.5-mm spacing for linear movement and 4.3° spacing for rotational movement, (d) a 5 × 5 array with 2-mm spacing for linear movement and 5.7° spacing for rotational movement, and (e) a 6 × 6 array with 1.5-mm spacing for linear movement and 4.3° spacing for rotational movement.

The HIFU focal spots were generated at 2 or 3 mm intervals (Figures 13(a), 13(b), and 13(d)) in a distinct 2D array pattern in the BSA phantom. These noncoalesced spots allowed us to accurately identify and analyze the 2D position of each HIFU spot. Scanning at 1.5 mm intervals showed the array pattern coalescing (Figures 13(c) and 13(e)). The nominal and actual positions of the HIFU focal spots are depicted in Figure 14(a) for the three array patterns corresponding to Figures 13(a), 13(b), and 13(d). The offset between the nominal and actual position is illustrated in Figure 14(b).

The root–mean-square error (RMSE) of the offsets between the nominal and actual positions is summarized in Table 4. The RMSE observed in the 2D array patterns is comparable to the positional accuracy obtained from only one-dimensional motion in each direction in the previous section. The 2D stepwise scanning also fulfills the focal positional accuracy requirement of our HIFU system in both the *X* and *Z* directions, achieving accuracy within the specified tolerance of 1 mm.

The article "Motion Accuracy of Pneumatic Stepper Motor-Driven Robotic System Developed for MRI-Guided High-Intensity Focused Ultrasound Treatment of Prostate Disease" was published in 2024. Journal: Appl Bionics Biomech.

## 4. Discussion

Ensuring the MRI compatibility of the entire HIFU system, including its actuator, is crucial for the safe and effective clinical application of MRI-guided HIFU treatment technology, where precise targeting and monitoring are paramount. The MRI compatibility test conducted on our prototype transrectal HIFU robotic system, utilizing pneumatic stepper motors, revealed a 2.8% decrease in SNR during motor operation. This observed decrease is comparable to or better than that reported in other pneumatic motor studies: Sajima et al. [16] reported an 11% SNR decrease, while Chen et al. [17] reported a 2.35% decrease. The SNR reduction in our system, though not significant, appeared to have been caused by the potentiometers operating inside the MRI bore, drawing a small amount of current. While this SNR reduction did not result in any noticeable noise in the MRI images, future research could investigate alternative options to mitigate potential noise interference from the potentiometers. For instance, exploring alternatives such as optical fiber-based encoders could further enhance MRI compatibility.

In crafting the robotic device, we prioritized dimensions and form factors that would accommodate for patients in the dorsal recumbent position on the MRI couch, thus guaranteeing clinical relevance. The device's width is noticeably narrower than the couch, facilitating the safe and easy placement of it onto the couch. We meticulously designed and developed a pneumatic stepper motor-driven HIFU robotic system with sufficient power to actuate the transducer. The prototype employed in this study was constructed from PLA utilizing a 3D printer. It effectively demonstrated the transducer actuation without encountering any issues such as deformation or damage to its components. As a prototype model, our primary objective was to validate positional accuracy and create HIFU focal spots in a 2D array within tissue-mimicking phantoms. To ensure long-term robustness and reliability, our next plans involve utilizing stronger 3D printing materials such as acrylonitrile butadiene styrene, polyethylene terephthalate glycol, polyamide, or polycarbonate for preclinical and clinical trials. If mass production becomes necessary in the future, injection molding may be considered for its cost-effectiveness. Maintaining a consistently stable air pressure input into the pneumatic system is crucial for ensuring reliable performance of pneumatic motors. In our study, we employed an air compressor and a pressure regulator. The air compressor generated loud acoustic noise during operation, and there is concern about the risk of microbiological contamination associated with supplying ambient room air into the compressor, potentially introducing bacteria and viruses into the compressed air system. Therefore, we are considering supplying nitrogen gas at a constant pressure instead of using an air compressor.

The article "Motion Accuracy of Pneumatic Stepper Motor-Driven Robotic System Developed for MRI-Guided High-Intensity Focused Ultrasound Treatment of Prostate Disease" was published in 2024. Journal: Appl Bionics Biomech.

While motion accuracy may depend on the load and input pressure applied to the pneumatic stepper motors, our HIFU system maintains consistent settings for both during the HIFU procedure. Our objective was to assess the anticipated precision of transducer positioning and positional accuracy of the focal spots generated during HIFU treatment for prostate disease. Therefore, the positional accuracy assessments were conducted under conditions that encompass factors such as input pressure, the length of the pneumatic tubes, and the transducer mounting inside the probe, identical to those encountered during actual HIFU procedures. The assessment pertains to Motors 1 and 2, while Motor 3 is irrelevant to the positional accuracy assessment, as it does not participate in the movement of the transducer during the HIFU procedure. The positional accuracy of the linear motion of the transducer actuated by the robotic device was measured to be ±0.20 and ±0.22 mm for the forward and backward directions, respectively, and the positional accuracy of the rotational motion was measured to be ±0.79° and ±0.74° for CW and CCW directions, respectively. These results demonstrated that the proposed system is suitable for clinical application. To the best of our knowledge, no specific specifications have been established for the mechanical positional accuracy of HIFU systems. According to the guidelines of the MFDS in South Korea, the HIFU focal spot positional accuracy should be within ±1 mm. When developing our robotic system, our aim regarding the positional accuracy of the transducer was to adhere to the guidelines outlined by the MFDS, ensuring alignment with regulatory standards. The measured positional accuracy of the transducer does not include deviations caused by incomplete calibration but is a combination of errors from the stopping accuracy of the pneumatic motor, motor step size, potentiometer resolution, and potentiometer linearity. We achieved our goal of positional accuracy of less than 1 mm in all directions. Additionally, we expect that utilizing high-resolution potentiometers or encoders will further enhance the positional accuracy.

The article "Motion Accuracy of Pneumatic Stepper Motor-Driven Robotic System Developed for MRI-Guided High-Intensity Focused Ultrasound Treatment of Prostate Disease" was published in 2024. Journal: Appl Bionics Biomech.

To ablate the target tumor in the prostate, usually one cubic centimeter or larger, a stepwise scanning approach is utilized at spatial intervals of several millimeters. As the transducer moves along scanning pathways, changes of direction occur multiple times, inevitably leading to positional errors caused by backlash. Backlash, defined as the clearance occurring in the direction of motion within mechanical devices that mesh with each other, such as screws and gears, is not inherently problematic as long as the gear pair maintains a consistent direction of rotation. However, issues arise when the gear changes its direction of rotation, resulting in a change in the contacting side of the teeth. As one gear's teeth approach the backlash space, it may rotate without exerting force on the other gear. Consequently, the gear with backlash rotates less, leading to positional errors in the actuator. In our robotic device, the gear shaft of the pneumatic stepper motor meshes with the spur gear of the probe for rotational motion and the probe's rack gear for the transducer's linear motion, introducing backlash into the system. Backlash posed a significant obstacle whenever the direction of movement of the transducer was reversed both in linear and rotational motions, resulting in substantial positional errors exceeding 1 mm (Figures 11(a) and 11(b)). To address this, we developed software compensation, effectively mitigating the large positional errors caused by backlash (Figures 11(c) and 11(d)). Although the software compensation for backlash worked effectively, it took more time for the transducer to move to the next point because additional movement and directional changes were required. Devising a backlash-free system could offer an alternative solution to the backlash problem. We envisage two methods to achieve such a system. First, attaching an encoder directly to the drive shaft of the transducer, bypassing the need for gears. Position control via a closed-loop feedback system utilizing an encoder eliminates positional errors arising from backlash. Second, constructing a system that utilizes a timing belt instead of directly meshing two gears. Timing belts and pulleys can be employed to develop systems devoid of backlash.

During HIFU treatment of prostate tumors, the stepwise scanning approach merges HIFU focal spots to create coalesced lesions within living tissue. By iterating the stepwise scanning process multiple times, the entire prostate can also be cauterized. In our study, this scanning and coalescing process was briefly emulated utilizing the BSA phantom, a well-established tissue-mimicking model in HIFU experiments. HIFU focal spots generated at 1.5 mm intervals exhibited coalescence (Figures 13(c) and 13(e)), whereas those generated at 2 or 3 mm intervals did not (Figures 13(a), 13(b), and 13(d)). By intentionally setting the HIFU focal spot size to 1.5 mm diameter, we aimed to precisely test positional accuracy in the BSA phantom under specific sonication parameters. Unlike conventional HIFU treatments for prostate cancer, which use 3 mm focal spots without spacing, we avoided coalesced lesions to ensure accurate measurement of individual focal spot positions. This allowed us to verify if the transducer motion accuracy with our robotic device translated to accurate focal spot positions within the BSA phantom. Our analysis revealed that the RMSE of offsets between nominal and actual positions ranged from 0.36 to 0.53 mm in the *X*-axis direction and from 0.19 to 0.31 mm in the *Z*-axis direction, both less than 1 mm (Table 4). This successful generation of 2D arrays of HIFU focal spots, achieving focal positional accuracy within 1 mm in the BSA phantom utilizing our developed HIFU robotic system, underscores its potential for inducing thermal ablation of desired sizes in various-sized tumors, particularly in prostate disease management.

The article "Motion Accuracy of Pneumatic Stepper Motor-Driven Robotic System Developed for MRI-Guided High-Intensity Focused Ultrasound Treatment of Prostate Disease" was published in 2024. Journal: Appl Bionics Biomech.

## 5. Conclusion

The prototype robotic system, employing MRI-compatible pneumatic stepper motors, has achieved clinically acceptable positional accuracy of the HIFU transducer movement within an intrarectal probe developed for MRI-guided HIFU treatment of prostate disease. Assessment confirmed MRI compatibility, with negligible distortion in MRI images and only a minor decrease in SNR during motor operation. The successful generation of 2D arrays of HIFU focal spots in tissue-mimicking phantoms demonstrates a capability easily adaptable to clinical requirements. Our findings suggest promising potential for future clinical applications of the robotic system in HIFU treatment. Future studies could involve in vivo experiments and clinical trials.

## Figures and Tables

**Figure 1:** Front (a) and back (b) views of MR-compatible transrectal HIFU probe housing transducer.

**Figure 2:** SolidWorks drawing for four-cylinder configuration within pneumatic stepper motor.

**Figure 3:** Developed pneumatic stepper motor with the four-cylinder configuration (a) and inside of planetary gearbox (b) coupled with motor.

**Figure 4:** Principle of converting the linear oscillating motions of the pistons into rotational motion of the geared axle through sequential pressure application, illustrating five sequential states labeled as (a) through (e).

**Figure 5:** Developed MR-compatible HIFU robotic system utilizing three pneumatic stepper motors viewed from top (a) and bottom corner (b).

The article "Motion Accuracy of Pneumatic Stepper Motor-Driven Robotic System Developed for MRI-Guided High-Intensity Focused Ultrasound Treatment of Prostate Disease" was published in 2024. Journal: Appl Bionics Biomech.

**Figure 6:** External robotic system controller developed to control transducer movement and HIFU firing at 5 m from MRI bore.

**Figure 7:** Experimental setup in the MRI scanner for assessing the MRI compatibility of the robotic device.

**Figure 8:** Experimental setup for irradiating HIFU into BSA phantom.

**Figure 9:** Zigzag raster scanning employed to generate a 2D array of HIFU focal spots, as illustrated by a 3 × 3 array example. The numbers indicate the scanning order, and the red arrow lines depict the trajectories of transducer motion. Stepwise scanning facilitates the fusion of HIFU focal spots into larger thermal lesions.

**Figure 10:** T1 GRE images of the axial plane under various activation conditions of the robotic device: (a) phantom only, (b) robot connected, and (c) robot in operation. The subtraction images (d, e) were derived by subtracting “robot connected” and “robot in operation” images, respectively, from the “phantom only” image.

**Figure 11:** Displacement error of transducer during stepwise scanning: (a) ten successive forward steps followed by ten successive backward steps along *Z*-axis with 3-mm step increments without backlash compensation, (b) while ten successive CW steps followed by ten successive CCW steps along *Φ*-axis with 8.6° step increments without backlash compensation. By contrast, (c, d) same motion as (a, b), respectively, but with backlash compensation.

**Figure 12:** Four error distributions, each derived from 40 samples: (a) the upper panel represents forward linear motion along the *Z*-axis with 3-mm step increments, while the lower panel represents backward linear motion along the same axis. (b) The upper panel illustrates CW rotational motion along the *Φ*-axis with 8.6° step increments, and the lower panel illustrates CCW rotational motion along the same axis. Error bars in each distribution represent statistical uncertainties. Gaussian functions were employed to fit each distribution and determine mean, SEM, and SD.

**Figure 13:** Five different array patterns formed in BSA phantom at plane perpendicular to HIFU beam: (a) 3 × 3 array with 2-mm spacing, (b) 3 × 3 array with 3-mm spacing, (c) 3 × 3 array with 1.5-mm spacing, (d) 5 × 5 array with 2-mm spacing, and (e) 6 × 6 array with 1.5-mm spacing.

**Figure 14:** Comparison between nominal and actual positions of the HIFU focal spots for three array patterns created in the BSA phantom: (a) the overlay of the nominal and actual positions and (b) the offset between the nominal and actual positions. Error bars in each plot represent the measured positional accuracies of the transducer movement.

The article "Motion Accuracy of Pneumatic Stepper Motor-Driven Robotic System Developed for MRI-Guided High-Intensity Focused Ultrasound Treatment of Prostate Disease" was published in 2024. Journal: Appl Bionics Biomech.

**Table 1:** SNR computed from the MRI images obtained under the three conditions.

Condition	Mean intensity	SD	SNR	Normalized SNR (%)
Phantom only	2,936.8	24.3	121.0	100.0
Robot connected	2,935.2	24.9	118.0	97.5
Robot in operation	2,931.4	24.9	117.7	97.2

**Table 2:** Positional accuracy of transducer in linear motion along *Z*-axis.

Direction	Linear error (mm)	
	Mean ± SEM	SD
Forward	0.00 ± 0.03	0.20
Backward	−0.13 ± 0.04	0.22

Mean, SEM, and SD were obtained from 40-time sampling error distribution.

**Table 3:** Positional accuracy of transducer in rotational motion along *Φ*-axis.

Direction	Angular error (°)	
	Mean ± SEM	SD
CW	0.18 ± 0.12	0.79
CCW	0.13 ± 0.12	0.74

Mean, SEM, and SD were obtained from 40-time sampling error distribution.

**Table 4:** RMSE of the offsets between the nominal and actual positions of the HIFU focal spots created in the BSA phantom.

Array	RMSE (mm)	
	*X*-axis direction	*Z*-axis direction
3 × 3 array with 2-mm spacing	0.36	0.31
3 × 3 array with 3-mm spacing	0.53	0.19
5 × 5 array with 2-mm spacing	0.52	0.20

## Data Availability

The data that support the findings of this study are available from the corresponding author upon reasonable request.
